# Clinical Study on the Efficacy of Laparoscopic Hepatectomy and Its Influence on the Expression of Serum VEGF, FGF, and Immune Function

This article has been retracted.

**DOI:** 10.1155/2021/4432022

**Published:** 2021-10-05

**Authors:** Zhengyong Tang, Yi Tang, Tianqi Liu, Rongjun Liu, Shaowei Xie, Dongyi Xie, Jianrong Yang, Yuntian Tang

**Affiliations:** Department of Hepatobiliary, Pancreas and Spleen Surgery, The People's Hospital of Guangxi Zhuang Autonomous Region, Guangxi Academy of Medical Sciences, Nanning, China

## Abstract

Liver cancer is one of the most common malignant tumors. Partial hepatectomy is the most basic and effective treatment for hepatocellular carcinoma because of its high operative effect and perioperative safety. Open surgery is the most traditional hepatectomy. Although it can completely remove tumor lesions and prolong patient survival, it has disadvantages such as large trauma and long postoperative recovery time. Meanwhile, long-term bed rest can increase the risk of complications such as venous thrombosis and infection. The advantages of laparoscopic partial hepatectomy, such as clear operative field, simple operation, little trauma, light surgical stress, quick postoperative recovery, and low complications, can avoid damage to vital organs, blood vessels, and nerves, which has been widely accepted and recognized in clinical practice.

## 1. Introduction

Liver cancer is one of the common malignant tumors in my country, with a high degree of malignancy, and the 5-year survival rate of patients is less than 8.5% [1, 2]. Since hepatocellular carcinoma has no specific symptoms in the early stage, patients often go to the doctor when the liver cancer ruptures and hemorrhages or when complications such as gastrointestinal bleeding occur [3, 4]. At present, surgical operation is the only clinical method that has the possibility of cure. For hepatocellular carcinoma that has not metastasized, radical surgery can achieve good results. Both open surgery and laparoscopic surgery are currently more commonly used surgical methods [5, 6]. Traditional laparotomy has the advantages of simple operation and clear vision, but its trauma, pain, postoperative complications, and slow recovery process [7, 8]. In recent years, with the progress of medical technology and surgical instruments, especially the increasingly mature technology of laparoscopic surgery, the advantages of small trauma, rapid postoperative recovery, and low complications are increasingly prominent, which greatly improve the prognosis and postoperative quality of life of patients with liver cancer [9, 10]. However, due to the laparoscopic surgical technology and the precision of the instruments are still in the development stage, whether it can replace the traditional open liver resection is still a certain controversy. Studies have pointed out that the recovery and survival time of early liver cancer after surgery are closely related to the body's immune function, which helps to resist tumors and resistance to drugs. The trauma of surgery can cause immune function suppression and lead to changes in certain serum biochemical indicators [11]. This study aims to explore the curative effect of laparoscopic liver cancer resection and analyze its influence on the body's immune function, inflammatory factors, and various immunoglobulin factors. The specific report is as follows.

## 2. Materials and Methods

### 2.1. Patients

A retrospective analysis of 102 patients with liver cancer admitted to the department of hepatobiliary surgery of our hospital from June 2016 to June 2017 was performed. Inclusion criteria were as follows: all patients met the diagnostic criteria for hepatocellular carcinoma [12], with TNM stages I-II and Child–Pugh grade A or B; primary liver cancer was confirmed by pathological biopsy/imaging; this is consistent with the indications for hepatectomy. Exclusion criteria were as follows: patients who had received other antitumor therapies such as chemoradiotherapy before surgery; patients with metastatic liver cancer and at the same time, biliary tract reconstruction, cholecystectomy, and other operations; severe diseases of the immune, blood, endocrine, or nervous systems; those with a survival period of <3 months; and those who fall off during the follow-up. According to different surgical methods selected by patients, they were divided into the control group (*n* = 43) and the observation group (*n* = 59). There was no statistically significant difference in general information between the two groups (*P* > 0.05), as given in Table 1.

### 2.2. Treatment Method

The control group underwent open hepatectomy; the patients were operated in supine position and were treated with general anesthesia. The incision was at the lower margin of the right rib. After opening, the situation around the liver was routinely explored, and the surrounding blood supply was blocked. Subsequently, the liver tumor lesions were resected, and the resection line should be consistent with the direction of scraping. When large blood vessels were encountered, they should be consistent with the direction of the blood vessels to avoid cutting. Electrocoagulation was performed on the wound to stop bleeding. After the operation, the incision was sutured routinely.

Patients in the observation group underwent laparoscopic hepatectomy; the patient was placed in a supine position with head high and feet low. During the operation, the position was adjusted according to the position of the tumor, general anesthesia was given, and the tracheal intubation was performed. The pressure was about 12–16 mmHg pneumoperitoneum by filling with CO_2_. The four-hole method is used to enter the abdomen for surgery. The main operation hole is close to the tumor lesion, and the other operation holes are fan-shaped distributed in the liver lobe where the liver is located. First, the whole abdomen was investigated for adhesion and other conditions under laparoscope, and the location and size of the tumor were determined. Then, the ligaments around the liver were severed with an ultrasonic knife, so that the liver was fully exposed to the operative field, and a pretangent line was made on the surface of the liver, with the incision margin more than 2 cm away from the tumor. After sufficient dissection of the bile ducts and blood vessels, the liver tumor was resected. The small blood vessels and bile ducts could be directly dissected, while the large blood vessels and bile ducts should be clipped and dissected. Intraoperative electrocoagulation was performed to stop bleeding. After the operation, the laparoscopic surgical instruments were taken out, the incision was sutured, and the abdominal drainage tube was indwelled.

Both groups were given conventional antiinfection, acid suppression, and liver protection treatments after surgery.

### 2.3. Observation Index

The operative time, intraoperative blood loss, hepatis porta block time, time to get out of bed, and hospitalization time were compared between the two groups. All patients were followed up for 1 year. The incidence of complications such as pulmonary infection, biliary leakage, urinary tract infection, incision infection, and abdominal infection in the two groups was compared, the survival and recurrence of the patients were recorded, and the survival and recurrence rates were calculated. The levels of peripheral blood T lymphocyte subsets such as CD3+, CD4+, and CD8+ were compared between 2 groups before and after operation. Serum levels of the vascular endothelial growth factor (VEGF), acidic fibroblast growth factor (aFGF), and basic fibroblast growth factor (bFGF) were compared between 2 groups before and after surgery. Serum immunoglobulin A (IgA), IgM, and IgG levels were compared between the two groups before and after surgery.

### 2.4. Detection Method

5.0 ml of fasting peripheral venous blood was extracted from the patients in the morning before and 3 days after surgery and separated in a 3000 r/min centrifuge for 10 min. Serum was separated and extracted. Serum VEGF, aFGF, bFGF, IgA, IgM, and IgG levels were detected by the enzyme-linked immunosorbent assay (ELISA) with the kit provided by Shanghai Jianglai Biotechnology Co., Ltd. The specific operation steps are strictly in accordance with the kit instruction. The levels of CD3+, CD4+, and CD8+ T cells in serum were detected by flow cytometry. The specific procedures were strictly according to the kit instructions. The instrument was purchased from Beckman Coulter Co., Ltd., in the United States.

### 2.5. Efficacy Evaluation Criteria

According to the response evaluation criteria in solid tumor v1.1 (RECIST v1.1) [13], the curative effect was evaluated, and the objective remission rate = (complete remission + partial remission + stable disease)/total number of cases × 100%.

### 2.6. Statistical Method

The results of this experiment were statistically analyzed by SPSS 20.0 (SPSS Co., Ltd., Chicago, USA). Count data were expressed by rate, and the chi-square test was used for their comparison between groups. Measurement data were expressed by mean ± standard deviation, and the *t* test was used for their comparison between groups. *P* < 0.05 indicates that the difference is statistically significant.

## 3. Results

### 3.1. Comparison of the Short-Term Curative Effect between Two Groups of Patients

In the control group, 24 cases had complete remission, 12 cases had partial remission, 3 cases had stable disease, and 2 cases had disease progression, with the objective remission rate as 95.35% (41/43). In the observation group, there were 36 cases of complete remission, 17 cases of partial remission, 2 cases of stable disease, and 2 cases of disease progression, with the objective remission rate as 96.61% (57/59). There was no statistically significant difference in the objective remission rate between the two groups (*P* > 0.05), as shown in Figure 1.

### 3.2. Comparison of the Surgical Effect Indexes of the Two Groups of Patients

There was no statistically significant difference in the operation time and hepatic portal block time between the two groups of patients (*P* > 0.05). The intraoperative blood loss, time to get out of bed, and hospitalization time in the observation group were lower than those in the control group (*P* < 0.05), as shown in Figure 2.

### 3.3. Comparison of Complications, Recurrence, and Survival of the Two Groups of Patients

In the control group, there were 2 cases of pulmonary infection, 1 case of incision infection, and 2 cases of abdominal cavity infection, with the total incidence of complications as 11.63% (5/43). In the observation group, 1 case of urinary tract infection occurred, with the total incidence of complications as 1.69% (1/59). The total incidence of complications in the observation group was lower than that in the control group (*P* < 0.05). There was no statistically significant difference in the recurrence rate and survival rate between the two groups after surgery (*P* > 0.05), as shown in Figure 3.

### 3.4. Comparison of the Levels of T Lymphocyte Subsets between the Two Groups of Patients before and after Surgery

There was no significant difference in serum CD3+, CD4+, and CD8+ levels between the two groups before surgery (*P* > 0.05). 3 days after surgery, the serum CD3+ and CD4+ levels of the two groups were lower than those before the operation, and the CD8+ levels were higher than those before the operation (*P* < 0.05). 3 days after surgery, the serum CD3+ and CD4+ levels of the observation group were higher than those of the control group, and the CD8+ level was lower than that of the control group (*P* < 0.05), as shown in Figure 4.

### 3.5. Comparison of Serum VEGF, aFGF, and bFGF Levels before and after Surgery between the Two Groups

There was no significant difference in serum VEGF, aFGF, and bFGF levels before surgery between the two groups (*P* > 0.05). 3 days after surgery, the serum VEGF, aFGF, and bFGF levels in the two groups were lower than those before the operation, and the observation group was lower than the control group (*P* < 0.05), as shown in Figure 5.

### 3.6. Comparison of Immunoglobulin Expression Levels between the Two Groups of Patients before and after Surgery

There was no significant difference in serum IgA, IgG, and IgM levels between the two groups before surgery (*P* > 0.05). 3 days after surgery, the serum IgA, IgG, and IgM levels of the two groups of patients were lower than those before the operation, and the observation group was higher than the control group (*P* < 0.05), as shown in Figure 6.

## 4. Discussion

Primary hepatocellular carcinoma (HCC) is a malignant tumor with high incidence, recurrence rate, and mortality rate. Up to 90.0% of HCC is hepatocellular carcinoma. Viral hepatitis B, C, and other viral hepatitis are important contributing factors for HCC, so it is difficult to be diagnosed with a long and hidden onset process and no specific symptoms and signs in the early stage [14, 15]. Studies [16] have shown that most of the patients with liver cancer in my country have progressed to the middle and advanced stages. At this time, hematological metastasis has occurred, portal vein cancer thrombus has appeared, and extrahepatic organs such as the lung, bone, adrenal gland, and brain have been violated. The five-year survival rate is still extremely low with comprehensive treatment programs such as radiotherapy and chemotherapy. In recent years, with the development of early screening for malignant tumors and the improvement of people's health awareness, the early diagnosis rate of liver cancer has increased significantly. Therefore, more and more patients have the opportunity of surgical resection to provide them with the possibility of radical treatment of the disease. The National Comprehensive Cancer Network (NCCN) guidelines for the diagnosis and treatment of hepatocellular carcinoma proposed that for early liver cancer with a tumor diameter of less than 5 cm or multiple tumors with a diameter of less than 3 cm and no local or distant metastasis, partial hepatectomy has a high surgical effect and perioperative safety and is its most basic and effective treatment plan [17]. Open hepatectomy is the most traditional hepatectomy. Although it can completely remove tumor lesions and prolong patient survival, it has disadvantages such as large trauma and long postoperative recovery time. Meanwhile, long-term bed rest can increase the risk of complications such as venous thrombosis and infection [18–20]. With the improvement of laparoscopic equipment and technical experience, laparoscopy in cholecystitis, appendicitis, disease such as surgical treatment for rectal cancer with extensive application, the clear operation field, easy operation, small trauma, surgical stress lightweight, fast recovery, and low complications advantages can avoid to vital organs, blood vessels, and nerve injury; now, it has been widely accepted and approved clinically [21–23].

Laparoscopic hepatectomy has been used for more than 20 years. In the early stage, due to immature instruments and techniques, as well as complex anatomical structure, it is difficult to carry out partial hepatectomy, leading to its relatively slow development. But at present, it has become the operative method with the highest application rate for early liver cancer [24, 25]. Due to the small trauma, less intraoperative bleeding, laparoscopic surgery can reduce the pain of patients, and patients can get out of bed after the operation and then can greatly reduce the occurrence of lung infection, urinary tract infection, incision infection, and other complications. According to a 2011 survey [26], the annual cases of laparoscopic hepatectomy in China accounted for 20.00% of the total cases in the world, ranking second only to 28.00% in the United States. Compared with traditional open surgery, its advantages of less trauma, faster postoperative recovery, and lower complications have been widely recognized. The results of this study showed that the intraoperative blood loss, time to get out of bed, and hospitalization time in the observation group were lower than those of the control group, and the total incidence of complications was lower than that of the control group. It shows that the surgical effect and safety of laparoscopic hepatectomy are better than that of open hepatectomy, which is basically consistent with the current reports [27].

Malignant biological indicators are an important criterion for evaluating the condition and prognosis of tumors. Studies [28] have pointed out that there are often differences in malignant biochemical indicators among patients with different surgical liver cancers. In this study, the author compared the immune function, inflammatory factors, and malignant biological indicators of the two groups of patients before and after surgery and aimed to study the correlation between the indicators and provide a more comprehensive basis for the selection of clinical surgery. Immunosuppression is considered to be an important factor affecting postoperative recovery and survival of early liver cancer. Psychological and physiological stress caused by surgical trauma can inhibit cellular immune function of the body, and the greater the trauma, the stronger the inhibition, which directly affects postoperative recovery. Studies have confirmed that humoral immunity can recognize tumor cell-specific antigens through the secretion of various antibodies by plasma cells, can activate complement to initiate the cell killing mechanism, and can effectively mediate the conditioning effect, which plays an important role in the body's antitumor. As the most important immunoglobulin in humoral immunity, IgG can specifically recognize antigens, activate the complement killing mechanism, and enhance the phagocytosis and killing effect of macrophages on tumor cells, while IgM can effectively activate complement-mediated phagocytosis and killing function of phagocytes, and IgA mainly plays a mucosal protection role. When the body is stimulated by stress or traumatic surgery, the content of immunoglobulin in the blood can be significantly reduced, humoral immune function is suppressed, and the degree of suppression is obviously positively correlated with trauma. The results of this study showed that the levels of serum IgA, IgG, and IgM in the observation group were significantly higher than those in the control group 3 days after surgery, indicating that laparoscopic surgery has less trauma and immune function suppression, which is beneficial for patients to recover after surgery. Compared with before the operation, the observation group's CD3+ and CD4+ 3 days after the operation decreased lower in the control group and the CD8+ increased lower than the control group, suggesting that laparoscopic surgery has less immune function suppression. The analysis of the reason is that the laparoscope adopts the laparoscopic lens and the instruments, which are guided by the laparoscopic lens to transmit the image to the information processing system, and the surgical operation is more precise. At the same time, the operation method of 2–4 holes is adopted, and the abdominal wall is pierced with 3–10 mm, which causes light damage to the abdominal wall, so as to reduce the suppression of immune function caused by the traumatic stress of surgery. VEGF is a highly specific provascular endothelial cell growth factor, which is highly expressed in a variety of malignant tumors and can promote neoangiogenesis of tumors. FGF is a factor promoting tumor focus formation, which can promote endothelial cell migration and smooth muscle cell proliferation, as well as promote tumor neoangiogenesis, and is an important malignant biological indicator of liver cancer [29, 30]. The results of this study showed that the serum VEGF, aFGF, and bFGF levels of the observation group were significantly lower than those of the control group 3 days after surgery. The analysis of the reasons is related to the light traumatic stress and inflammatory stress of laparoscopic surgery and the small immunosuppressive effect on the body, but the exact factors still need to be further studied.

## 5. Conclusion

Laparoscopic hepatocellular carcinoma resection has the advantages of small trauma, low blood loss, and low complications in the treatment of hepatocellular carcinoma. At the same time, it has light inhibition on the immune function of the body and can reduce the expression of serum malignant biological indicators, which is worthy of clinical promotion.

## Figures and Tables

**Figure 1:** Comparison of the short-term curative effect between two groups of patients.

**Figure 2:** Comparison of the surgical effect indexes of the two groups of patients. Compared with the control group, ^*∗*^*P* < 0.05.

**Figure 3:** Comparison of complications, recurrence, and survival of the two groups of patients. Compared with the control group, ^*∗*^*P* < 0.05.

**Figure 4:** Comparison of the levels of T lymphocyte subsets between the two groups of patients before and after surgery. Compared with before surgery, ^*∗*^*P* < 0.05. Compared with the control group, ^#^*P* < 0.05.

**Figure 5:** Comparison of serum VEGF, aFGF, and bFGF levels before and after surgery between the two groups. Compared with before surgery, ^*∗*^*P* < 0.05. Compared with the control group, ^#^*P* < 0.05.

**Figure 6:** Comparison of immunoglobulin expression levels between the two groups of patients before and after surgery. Compared with before surgery, ^*∗*^*P* < 0.05. Compared with the control group, ^#^*P* < 0.05.

**Table 1:** Comparison of two general data.

Groups	Sex		Age (years old)	Tumor diameter (cm)	Child–Pugh classification		TNM staging	
	Male	Female			A	B	I	II
Control group (*n* = 43)	28	15	58.44 ± 12.65	3.38 ± 0.92	34	9	20	23
Observation group (*n* = 59)	33	26	59.63 ± 13.25	3.26 ± 1.02	40	19	28	31
*t/χ* ^*2*^	0.873		0.456	0.611	1.587		0.009	
*P*	0.351		0.649	0.543	0.208		0.925	

## Data Availability

The data used to support the findings of this study are available from the corresponding author upon request.
